# Correlation Analysis between the Emotion and Aesthetics for Chinese Classical Garden Design Based on Deep Transfer Learning

This article has been retracted.

**DOI:** 10.1155/2022/1828782

**Published:** 2022-07-09

**Authors:** Bao Guanglong, Gao Qian

**Affiliations:** College of Fine Arts and Design, YangZhou University, Yangzhou 225000, Jiangsu, China

## Abstract

Garden design with healthy psychological characteristics is a design method that mines positive psychological expressions and converts them into garden design elements. Chinese classical gardens are cultural heritage of China. Studying the beauty of space in classical gardens is of great significance to inheriting traditional culture, traditional art, and traditional aesthetics. At present, the research hotspots of garden design with healthy psychological characteristics mainly focus on the construction of relevant research theories and methods with the help of various intelligent tools. In this study, we propose a deep learning-based end-to-end model to recognize the positive psychological design of a Chinese classical garden. The model is designed based on Inception V3 that is proposed by Google. The innovation lies in that transfer learning which is integrated into Inception V3 to improve the generalization ability. Also, it is not necessary to encode the characteristics of the garden design style due to the end-to-end structure used in our proposed model. We design a positive psychological characteristics classification task to recognize high aesthetic feeling and low aesthetic feeling of rockery design. Experimental results indicate that our proposed model wins the best performance compared with other comparison models.

## 1. Introduction

Chinese classical gardens refer to Chinese landscape gardens represented by private gardens in the south of the Yangtze River and royal gardens in the north, which are unique in the history of garden development in the world [1–5]. Chinese classical gardens are cultural heritage of China. Studying the beauty of space in classical gardens is of great significance to inheriting traditional culture, traditional art, and traditional aesthetics. Many concepts generated in the space of Chinese classical gardens, such as virtual reality, artistic conception, form, and the changes in people's aesthetic psychology caused by the viewer's aesthetic view and appreciation of the garden, are all important issues in aesthetics. The study of these issues is not only necessary for classical aesthetics but also concerned by modern aesthetics. As a kind of plastic art, gardens use individual landscape elements such as landscapes, plants, and buildings in the form of a community with a certain spatial combination relationship, presenting a variety of formal beauty and twisted, imitating the natural beauty of nature. The beauty of rhythm and sense of rhythm displayed by Chinese classical gardens in the construction of space have the same effect of educating people's hearts as music.

Garden design with healthy psychological characteristics is a design method that mines user psychological information and converts it into garden design elements [6–8]. At present, the research hotspots of garden psychological design mainly focus on the construction of relevant research theories and methods with the help of various intelligent tools. The design process is generally divided into three steps. First, user's psychological information is obtained and quantitatively represented. Secondly, the complex relationship between the user's psychological characteristics and the elements of garden design is established through a mapping model. Finally, the model is converted into an objective function and optimized by intelligent algorithms, so as to help designers quickly generate, reasonably evaluate, and optimize the design, which meets the user's psychological requirements.

For example, Guo et al. [9] used a neural network to build a product image evaluation model under the theoretical framework of Kansei Engineering and used a genetic algorithm to design and optimize the model to generate a product design scheme that meets the needs of users' psychological imagery. Zhao et al. [10] used a BP (back propagation) neural network to build a multiobjective evaluation model to complete the evaluation of the product image and then used the bee colony algorithm to optimize the model to help designers get a color scheme with better evaluation results. Guoshu et al. [11] proposed a design method that combines color scheme reuse and perceptual imagery. Firstly, the fuzzy processing technology was used to extract the color combination scheme from the source image, and then the interactive genetic algorithm was used to complete the fitness evaluation of the color scheme population, so as to obtain the product design scheme that meets the user's perceptual needs. Ding et al. [12] established a multidimensional psychological product design model using grey theory and other methods to solve the problem of multidimensional psychological demand in product design. They used a nondominated sorting multiobjective optimization algorithm to optimize the design and finally built an intelligent design system based on this method. It can quickly generate a design scheme that meets the needs of users' multidimensional psychological imagery.

The above studies provide research methods and intelligent tools for garden psychological design and effectively improve the quality of garden design. However, there are still some limitations in solving strategies. For example, on the one hand, during the research process, it is necessary to encode the characteristics of the garden design style and then build a correlation model between the features and the user psychological characteristics, and intelligently solve and decode the parameters of the correlation model based on artificial intelligence algorithms. Such a design process is rather cumbersome. On the other hand, the design scheme is obtained according to the evaluation criteria of the association model. The quality of the scheme completely depends on the accuracy of the model, and it is difficult to learn the implicit design rules directly from the samples, which weakens the diversity and innovation of the design scheme to a great extent. Recently, deep learning-based methods have been widely used in various fields. For example, Wang et al. proposed a classifier based on Inception V3 for pulmonary image classification [13]. Alotaibi et al. proposed a hybrid deep ResNet (residual neural network) and inception model for hyperspectral image classification.

Therefore, in this study, we propose a deep learning-based end-to-end model to recognize the psychological design of Chinese classical garden. The model is designed based on Inception V3 that is proposed by Google. The innovation lies in that we integrate transfer learning into Inception V3 to improve the generalization ability of our model. Also, it is not necessary to encode the characteristics of the garden design style due to the end-to-end structure used in our model. The following sections are organized as follows. In section 2, we will introduce our data set and methods. In section 3, we will report our experimental results and discuss them. In the last section, we will conclude our study and indicate the future study.

## 2. Correlation Analysis between the Emotion and Aesthetics

### 2.1. Data

We employed 20 students from Yangzhou University to collect 1000 rockery design images of different types from the Baidu gallery (https://image.baidu.com).  Figure 1 shows a toy example of selected rockery design images. 15 landscape architects are invited to conduct subjective aesthetic evaluation on these collected rockery design. Landscape architects calibrated all the images from three aspects of high aesthetic feeling, low aesthetic feeling, and uncertainty according to the guideline shown in Figure 2. When the psychological evaluation labels with eight or more participants were the same, this label was determined as the final label of the pattern. After removing the uncertain labels, we finally obtained labeled 700 rockery design images.

### 2.2. Methods

#### 2.2.1. Inception V3

The Inception model has been proposed by Google since 2014, which effectively avoids the contradiction between the network depth and accuracy requirements and structural performance saturation and ensures that the computational structure of the model and the dependence on hardware configuration are reduced without reducing the classification accuracy [14–16]. The Inception model provides a good solution for object classification tasks [13, 17, 18].

In this study, we employ Inception V3 as our psychological classification model. The network structure is shown in Figure 3. We also use the following techniques to improve the performance of Inception V3.

(1) LSR (least square regression) is used to reduce the overfitting problem. To be specific, we use *q*(*k*/*x*) to train Inception V3 in a manner of independent hot coding, and the output is the predictive probability distribution *p*(*k*/*x*) of normalized softmax function, where *p*(*k*/*x*) can be defined as follows:
  (1) $$\begin{array}{c} p\left(\frac{k}{x}\right)=\frac{e^{z_{k}}}{\sum_{i=1}^{k}e^{z_{k}}}, \end{array}$$
where the loss function can be defined as
  (2) $$\begin{array}{c} H\left(q,p\right)=\sum_{k=1}^{k}\log\left(p\left(k\right)q\left(k\right)\right). \end{array}$$
In order to solve the overfitting problem, Inception V3 adds weights to a certain probability distribution to form new labels. Specifically, the processing way can be mathematically expressed as
  (3) $$\begin{array}{c} q^{\prime }\left(\frac{y}{x}\right)=\left(1-a\right)q\left(\frac{y}{x}\right)+au\left(y\right), \end{array}$$
  (4) $$\begin{array}{c} q^{\prime }\left(\frac{y}{x}\right)=\left(1-a\right)q\left(\frac{y}{x}\right)+aK. \end{array}$$
In (3) *a* ∈ (0,1). Therefore, the loss function can be updated as
  (5) $$\begin{array}{c} H\left(q^{\prime },p\right)=-\sum_{k=1}^{k}\log\left(p\left(k\right)q^{\prime \left(k\right)}\right)=\left(1-a\right)H\left(q,p\right)+aH\left(u,p\right). \end{array}$$
(2) To reduce complexity, we use the convolution kernels of 1 × *n* and *n* × 1 to replace *n* × *n*.
(3) In the full connection layer, we adopt the batch-normalization strategy.
(4) The RMSProp (root mean squared propagation) optimization strategy is employed to make the proposed structure which has the ability of self-adaptative learning, that is,
  (6) $$\begin{array}{c} \left\{\begin{array}{c} \text{d}w_{i}=\frac{\text{d}L\left(w\right)}{\text{d}w_{i}},\\ S\text{d}w_{i}=\rho S\text{d}w_{i}+\left(1-\rho \right)\text{d}w_{i}^{2}, \end{array}\right. \end{array}$$
  where *ρ* is the attenuation coefficient.

#### 2.2.2. Transfer Learning

In this study, owning to the small size of the training set, we introduce transfer learning to learn extra knowledge from the public dataset so as to assist our model training [19, 20]. The flowchart of Inception V3 combining with transfer learning is shown in Figure 4. In Figure 4, the ImageNet dataset is taken as the source domain, and Inception V3 without full connection and softmax layers are used to extract deep features from the source domain, then the deep features are taken as transfer knowledge to guide learning of our training data.

## 3. Experimental Studies

### 3.1. Settings

To evaluate the performance of our proposed model, we introduce three extra models, i.e., GoogleNet [21–25], ResNet [26–28], and VGG [29–32] for comparison. For all models, the learning rate is set to 0.0001, Adagrad is adopted as the optimizer [33–35], the upper bound of iteration is to set 200, the batch size is set to 32, and ReLU is selected as the activation function [36–38]. All training images are cropped into 224 × 224 × 3. Our experiments are conducted on a PC with Core™ i5-11400 Processor (12 M Cache, up to 4.40 GHz), RTX 2090 Ti 11G, and 32G memory.

### 3.2. Experimental Results and Discussions

Figure 5 illustrates the performance in terms of accuracy and loss for the four models where the *x*-axis represents the iterations, and the *y*-axis represents the performance in terms of accuracy. As can be seen from Figure 5, the four models perform well in terms of accuracy, gradually enter the convergence area after about 100 iterations, and maintain an accuracy rate of more than 90% and a loss function value below 0.5. The initial Inception V3 did not show significant advantages in terms of accuracy and loss. The accuracy of Inception V3 is not as good as VGG, but its convergence rate has obvious advantages, and it enters the 10% error band after 10 iterations.

It can be seen from Table 1 that the Inception V3 model combined with transfer learning (Transfer-Inception V3) performs well. The introduction of transfer learning effectively improves the learning starting point of the training model. Compared with VGG, the accuracy of Transfer-Inception V3 is improved by 0.0275. In terms of the convergence rate, Transfer-Inception V3 achieved around 0.9 accuracy after 30 to 40 iterations, while Inception V3 and VGG achieved around 0.9 accuracy after 100 and 80 iterations, respectively. In terms of recognition accuracy, Transfer-Inception V3 has been iteratively trained for 200 times, and the accuracy is basically stable around 0.98, while Inception V3 and VGG are around 0.92 and 0.95, respectively. Therefore, Transfer-Inception V3 performs better than Inception V3 and VGG in terms of the convergence rate and accuracy.

Transfer-Inception V3 and Inception V3 are further compared in terms of accuracy and loss, and the comparison results are shown in Figure 6. As can be seen from Figure 6, Transfer-Inception V3 well inherits the fast convergence of the initial Inception V3 and further optimizes the learning rate and loss of features. The initial value of Transfer-Inception V3 is better, and the accuracy tends to be smoother. Compared with the 0.92 accuracy of Inception V3, the learning rate of Transfer-Inception V3 is increased by 6% to 98%, and the corresponding loss is reduced to 0.06, which leads to an increase of about 70%. This further shows that in the problem of pattern recognition, transfer learning still has good inheritance and adaptability.

## 4. Conclusions

Chinese classical gardens are cultural heritage of China. Garden design with healthy psychological characteristics is a design method that mines positive psychological expressions and converts them into garden design elements. Studying the beauty of space in classical gardens is of great significance to inheriting traditional culture, traditional art, and traditional aesthetics. Garden psychological design is a design method that mines user's psychological expressions and converts them into garden design elements. In this study, we propose a deep learning-based end-to-end model to recognize the psychological design of the Chinese classical garden. The model is designed based on Inception V3 that is proposed by Google. Transfer learning is integrated into Inception V3 to improve the generalization ability. Also, it is not necessary to encode the characteristics of the garden design style due to the end-to-end structure used in our proposed model. We design a psychological classification task to recognize high aesthetic feeling and low aesthetic feeling of rockery design. Experimental results indicate that our proposed model wins the best performance compared with other comparison models. In the following work, we will expand the application scope of the proposed method in the emotional design of classical gardens.

## Figures and Tables

**Figure 1:** Example of selected rockery design images (https://image.baidu.com).

**Figure 2:** Guideline for psychological labeling.

**Figure 3:** The network structure of Inception V3.

**Figure 4:** The flowchart of Inception V3 combined with transfer learning.

**Figure 5:** Comparison of results in terms of accuracy and loss against iterations. (a) Accuracy. (b) Loss.

**Figure 6:** Transfer-Inception V3 vs. Inception V3 in terms of accuracy and loss against iterations. (a) Accuracy. (b) Loss.

**Table 1:** Performance of Transfer-Inception V3, Inception V3, and VGG in terms of accuracy.

Iterations	Transfer-Inception V3	Inception V3	VGG
1	0.6274	0.4678	0.3024
10	0.8345	0.8071	0.6328
20	0.8642	0.8075	0.7896
30	0.8971	0.8367	0.8444
40	0.9111	0.8487	0.8621
50	0.9261	0.8610	0.8569
60	0.9220	0.8887	0.8675
70	0.9421	0.8700	0.8721
80	0.9356	0.8804	0.9008
90	0.9567	0.8675	0.9141
100	0.9587	0.8976	0.9120
110	0.9614	0.9172	0.9170
120	0.9681	0.9150	0.9155
130	0.9682	0.9231	0.9289
140	0.9675	0.9247	0.9394
150	0.9876	0.9227	0.9321
160	0.9814	0.9234	0.9346
170	0.9811	0.9112	0.9345
180	0.9781	0.9243	0.9238
190	0.9872	0.9231	0.9452
200	0.9786	0.9231	0.9511

## Data Availability

The dataset can be accessed upon request.
